The article "Detecting Buildings and Nonbuildings from Satellite Images Using U-Net" was published in 2022. Journal: Comput Intell Neurosci.

# Detecting Buildings and Nonbuildings from Satellite Images Using U-Net

**DOI:** 10.1155/2022/4831223

**Published:** 2022-05-05

**Authors:** Waleed Alsabhan, Turky Alotaiby, Basil Dudin

**Affiliations:** ^1^Al Faisal University, College of Engineering, P.O.Box 50927, Riyadh 11533, Kingdom of, Saudi Arabia; ^2^King Abdulaziz City for Science and Technology, National Center for Artificial Intelligence, P.B. Box 6086, Riyadh 11442, Saudi Arabia

## Abstract

Automatic building detection from high-resolution satellite imaging images has many applications. Understanding socioeconomic development and keeping track of population migrations are essential for effective civic planning. These civil feature systems may also help update maps after natural disasters or in geographic regions undergoing dramatic population expansion. To accomplish the desired goal, a variety of image processing techniques were employed. They are often inaccurate or take a long time to process. Convolutional neural networks (CNNs) are being designed to extract buildings from satellite images, based on the U-Net, which was first developed to segment medical images. The minimal number of images from the open dataset, in RGB format with variable shapes, reveals one of the advantages of the U-Net; that is, it develops excellent accuracy from a limited amount of training material with minimal effort and training time. The encoder portion of U-Net was altered to test the feasibility of using a transfer learning facility. VGGNet and ResNet were both used for the same purpose. The findings of these models were also compared to our own bespoke U-Net, which was designed from the ground up. With an accuracy of 84.9%, the VGGNet backbone was shown to be the best feature extractor. Compared to the current best models for tackling a similar problem with a larger dataset, the present results are considered superior.

## 1. Introduction

The observation of the composition of structures in rural regions is critical to rural development [1]. Unplanned and insufficiently recorded homes, on the other hand, have provided considerable obstacles to comprehending rural communities [2, 3]. Field surveys have generally been the main option, but they demand a lot of effort and can be time-consuming, particularly in distant places. Recent advances in remote sensing technology have resulted in an increase in the provision of high spatial data photographs such as low-altitude aerial shots and unmanned aerial vehicle (UAV) photographs. Manual mapping of rural communities is now possible at a lower cost and with larger coverage, although it is still time-consuming. As a result, a robust, smart, and image-based system for mapping rural human settlements is urgently required. The work is critical since building maps give fundamental information for a variety of applications such as advertising, urban administration, and popularity estimation. In recent times, the ability to detect new buildings straight from satellite photos is especially helpful in zones where people move fast (due to nomadic, displaced, or relocating communities), as well as in remote locations where data collection of these new buildings is often performed arduously by hand and speedily obsolete. Satellite photos may also be used to analyze building damage after a natural catastrophe, providing for the design of an appropriate response in specific locations. Lastly, they might be quite useful for solar panel producers who wish to assess the potential roof surface in a certain location.

The article "Detecting Buildings and Nonbuildings from Satellite Images Using U-Net" was published in 2022. Journal: Comput Intell Neurosci.

As metropolitan regions feature buildings of unusual construction and proximity, contemporary research in the sphere of automated building extraction, aerial, and satellite photos are employed. Aerial and satellite imagery are the main sources of accurate and trustworthy geographical data. Satellite photos can provide useful information about the supplied urban environment scenarios. Satellite photos are aerial photographs shot at a proper height from the sky towards the ground [4]. For decades, constructing maps using remote sensing has been a major study area [5–9].

This study addresses the wider issue of semantic segmentation of satellite pictures by categorizing each image as relating to or not belonging to a building; however, there are several difficulties in pixel categorization of satellite photos. In general, picture segmentation confronts various challenges, one of the most difficult being the ability to educate on one database and generalize successfully on another. This is especially noticeable in satellite photos, as photographs in the test set may be subjected to variable lighting or even relate to different places than images in the training set.

Most traditional building categorization methods are mainly based on life experiences and artificial design characteristics such as morphological features of the residences, texture features, building and shadow companions, building spacing, and the topological correlations between buildings and roads [5, 10–12]. These procedures have reached a certain level of accuracy, but they are insufficient. Deep learning has had a significant impact on computer vision research in recent years [13]. Since deep learning arose and gained popularity in computer vision studies, it stimulated the growth of neural network designs like CNNs and their application to creating division [14, 15]. Convolutional neural networks (CNNs) perform very well in building detection tasks [16–20].

The article "Detecting Buildings and Nonbuildings from Satellite Images Using U-Net" was published in 2022. Journal: Comput Intell Neurosci.

We created a convolutional neural network inspired by the U-Net for this objective [21]. On a collection of two-dimensional satellite pictures, we trained our algorithm. The accompanying labels were binary masks or two-dimensional arrays with ones for pixels containing a building and zeros for those that did not. Using a satellite picture as input, our program was able to generate a projected binary mask. The U-Net design increases picture segmentation performance, although it is still insufficient for many purposes. Transfer learning is utilized to obtain the needed accuracy. To increase picture classification accuracy, ResNet and VGGNet encoders were added to the U-Net architecture. This obtained good results in medical picture categorization. We are attempting to study how transfer learning affects U-Net performance in this effort. This paper attempts to use U-Net with two distinct encoders, ResNet and VGGNet, to a remote sensing image classification assignment for building extraction and compares the reliability of the two approaches to the base model.

The major contributions of the works are as follows:

1. The work creates a computationally efficient and accurate model that will aid in the segmentation of buildings from satellite imagery
2. The current work develops a semantic segmentation model with a minimal number of images compared to previous works in the domain
3. The generated model outperforms prior models built with huge datasets in the same domain in terms of accuracy
4. The model is trained on RGB photos to take use of the different deep learning frameworks available for the intended task

The rest of the paper is laid out as follows: Section 2 reviews the current research problem's most recent and significant research.  Section 3 explains the datasets and architectures used in this study.  Section 4 discusses the findings, and the paper is concluded in Section 5.

## 2. Literature Review

Image segmentation for automated building recognition in satellite photos is a relatively new area of study. In this regard, just a few articles have been written on the subject. Several techniques for extracting things such as buildings or roads from aerial or high-definition satellite photos have already been suggested [22]. Reference [23] introduced an automatic building detection method based on ANN (artificial neural networks) that makes use of structural and spectral data from high-resolution satellite pictures. Reference [11] provides a probabilistic approach that leverages local feature vector extraction to conduct building extraction. The author identified spatial coherence as a set of joint random variables for building detection. The author considers four local feature extractions for estimating the probability density function. Other local feature extractions were also mentioned by him. For further improving building identification, two fusion approaches are implemented, one at the data level and the other at the classification stage. The author then related the building detection approach to the theory of spectral graphs. Support vector machine (SVM) methods were utilized in several publications to extract buildings from very high-resolution (VHR) satellite pictures [20, 24, 25]. In each example, the base-case accuracy is 74 percent and 83 percent, respectively.

The article "Detecting Buildings and Nonbuildings from Satellite Images Using U-Net" was published in 2022. Journal: Comput Intell Neurosci.

Recent research efforts have focused on using the convolution neural network (CNN) for good-quality satellite picture labeling. Nevertheless, obstacles remain determining the ideal CNN design for the best answer to such situations. Reference [14] produced 340 km^2^ of building segmentation datasets in Massachusetts and educated the CNN model for building categorization. Reference [26] suggested a multilayer perceptron strategy for creating labels to equalize the trade-off between localization and categorization. Reference [20] tackled the difficulty of retaining semantic segmentation borders in high-resolution satellite data by developing a novel spiraled multitask loss and considering the border space in consideration. In addition to developing new structures, researchers combined data from other sources. Reference [27] used edge detection data to generate clear class boundaries for building extraction. Reference [28] studied the use of OpenStreetMap (OSM) data to build a coarse to fine remedy for semantic tagging of satellite pictures.

Inria recently offered a suitable dataset for working on satellite photos, including training and validation images covering various geographic areas [29]. They also provide segmentation performance using a fully convolutional network (FCN) and its extension utilizing a multilayer perceptron [30].

Deep learning approaches have recently demonstrated great detection performance for building detection [31, 32]. However, the majority of deep learning systems devised does not segment buildings but rather detect them from satellite imagery. Several studies suggest semantic segmentation algorithms for creating segmentation [33]. They worked with a U-Net [21] and DeepLabv3+ [34]. The U-Net is utilized for building recognition in a variety of different works [35–39]. Reference [40] used the U-Net model to separate five different types of buildings using satellite pictures. Reference [41] employed the Mask R-CNN [42] method to obtain each version of the structure individually. Reference [43] used the similar strategy to separate ancient and new building types.

The article "Detecting Buildings and Nonbuildings from Satellite Images Using U-Net" was published in 2022. Journal: Comput Intell Neurosci.

## 3. Materials and Methods

### 3.1. Dataset Preparation

We have used the open dataset from [43] which was a modification of high-resolution satellite pictures of rural Xinxing County, Guangdong Province, China. The dataset consists of 68 images with a resolution of 0.26 m. All the images were in RGB color space and of varying size from 900 × 900 to 1024 × 1024. All the gathered images were already manually segmented and annotated using the VGG Image Annotator (VIA) [44] into 3 classes (background, new building, and old building). Of the total 68 images, only 34 images were only annotated as new and old building classes. As this number did not seem sufficient for our work, we limited the number of classes into two (nonbuilding and building). Also, the already existing dataset was particularly created for instance segmentation. But, our aim was to create a semantic segmentation on the collected images, where instead of specifying the coordinates of the bounded polygons corresponding to each class, we need pixel-wise labeling, so the segmentation masks and annotations in .json format were converted into the format suitable to train the semantic segmentation model.

The complete dataset was divided into training, validation, and test groups. The 54 images were allocated for training, 8 images for validation, and 6 images for testing. The corresponding annotation mask for each image was a binary mask where intensity value 0 for the pixels corresponded to the nonbuilding class and intensity value of 1 for the building class.  Figure 1 shows the sample images and corresponding annotations from the training, validation, and test dataset.

#### 3.1.1. Data Augmentation

Even though U-Net [21] successfully operates on a small number of training instances, we used real-time data augmentation techniques to our training set to preserve a suitable number of images. The collected satellite photos were rotated, flipped, zoomed, and sheared so that the training would be on a more extensive set of datasets and reduce overfitting. There is not much memory utilization as the data enhancement is done by the Keras [45] framework in real time while loading the batches for training.

### 3.2. Methodology

#### 3.2.1. Network Architecture

The process of image examination to find discriminative properties of objects of interest is known as image interpretation. Several stages are required to gain a complete comprehension of a scene from an aerial photograph. A segmentation stage divides a scene into sections of certain categories given an image, allowing the complete visual environment to be seen as a corresponding image of all categories. The process of grouping segments of photographs so that each pixel in a group matches the object class of the group as a whole is known as semantic segmentation [21, 46]. The object classes in this work match buildings and nonbuildings (background). The rest of this paper takes a deep neural network approach to the problem of segmenting satellite pictures, which has had a lot of success in recent years on image identification tasks.

The article "Detecting Buildings and Nonbuildings from Satellite Images Using U-Net" was published in 2022. Journal: Comput Intell Neurosci.

#### 3.2.2. U-Net

U-Net [21], as shown in Figure 2, is a U-shaped convolutional network, whose design is inspired from the traditional autoencoder. The encoder-decoder architectural design is used to overcome loss of features while encoding into low-dimensional space.

### 3.3. Contraction Path

The left side of the architecture is a contracting path, which is designed for feature extraction to achieve image classification. It consists of two 3 × 3 convolutional layers followed by a ReLU activation layer and a 2 × 2 maxpooling operation. In between two convolutional layers, a drop-out layer is present to prevent overfitting and coadaptation while learning the parameters. The learning only takes place at the convolution layers to present at the encoder side. The maxpooling layer contributes to the significant amount of reduction in the size of feature vectors. The doubling of the number of filters while moving from the top to bottom blocks helps to extract advanced features from the input image compromising the image resolution. Consequently, the location information of such features is lost.

#### 3.3.1. Bottleneck

This part of the network is between the contracting and expanding paths. The bottleneck is built from simply 2 convolutional layers (with batch normalization) with drop-out.

### 3.4. Expansion Path

The right side of the architecture is an expansion path, which decodes the output of the contraction path and retrieves segmentation maps of the image. A 2 × 2 upconvolution or transpose-convolution layer is employed to achieve the reverse of the convolution that happened in the previous layers to resume the original image maintaining the connectivity among patterns. At each block, transpose convolution followed by two 3 × 3 convolutions helps in extracting complex features by increasing the size of feature maps; however, their localization is not taken care of. With a focus on this issue, the feature map from the encoder side is cropped and concatenated to the corresponding blocks at the decoder side. Therefore, information on the relationship between neighborhood pixels, otherwise called contextual features, will be given from the contraction to the expansion path. Thus, a better learning of the features will take place along with their localization information to draw accurate segmentation boundaries for objects in the image. Consequently, these skip connections help to recover all those fine grain features that were lost during the downward transfer at the encoder side. A drop-out layer is also present between the convolution layers to avoid overfitting. A 1 × 1 convolution occurs at the last layer to achieve as many feature maps as the number of object classes we need to detect. The max-pooling operation aims to reduce the size of feature vectors and is absent at this decoding side as our aim is the actual image with segmentation boundaries around targeted objects.

The article "Detecting Buildings and Nonbuildings from Satellite Images Using U-Net" was published in 2022. Journal: Comput Intell Neurosci.

#### 3.4.1. Environment for Training

The U-Net architecture and the entire semantic segmentation technique were mainly built using the Keras [45] framework, backed by TensorFlow [47] and written in *Python*. NumPy, OpenCV, Scikit-Learn [48], and other open-source modules were used for all other processing and analysis. All the images were resized to 512 × 512 before feeding into U-Net for training. The training was carried out on a 32 GB NVIDIA Quadro P1000 GPU. With a learning rate of 0.001, we employed the Adam algorithm [49] for gradient-based stochastic optimization of objective functions. For both the training and validation datasets, we trained the model to 50 epochs with a batch size of two. The block diagram for the entire U-Net training is summarized in Figure 3. The trained model is applied on the test images to validate the performance of the model.

#### 3.4.2. Performance Evaluation

The performance measures were derived from the test dataset's confusion matrix.

True positives (TP): true positives occur when a data point's actual and expected classes are the same (both are positive).

True negatives (TN): these are situations in which the actual and expected classes are the same (both are negative).

False positives (FP): false positives occur when a data point is incorrectly classified into a class.

False negatives (FN): false negatives occur when a data point is incorrectly classified as not belonging to a class. Some of the other performance evaluation metrics are given in the form of the following equations:

(1) $$\begin{array}{c} \text{Accuracy}=\frac{TP+TN}{TP+TN+FP+FN}. \end{array}$$

(2) $$\begin{array}{c} \text{Recall}=\frac{TP}{TP+FN}. \end{array}$$

(3) $$\begin{array}{c} \text{Precision}=\frac{TP}{TP+FP}. \end{array}$$

(4) $$\begin{array}{c} \text{F}1\text{ score}=\frac{2*\text{Recall}*\text{Precision}}{\text{Precision}+\text{Recall}}. \end{array}$$

(5) $$\begin{array}{c} iOU=\frac{\text{TP }}{\text{TP}+\text{FP}+\text{FN }}. \end{array}$$

(6) $$\begin{array}{c} Dice=\frac{2*TP}{\left(TP+FP\right)+\left(TP+FN\right)}. \end{array}$$

The article "Detecting Buildings and Nonbuildings from Satellite Images Using U-Net" was published in 2022. Journal: Comput Intell Neurosci.

## 4. Results and Discussion

We began by constructing a basic U-Net architecture, similar to that proposed in reference [21], but without any train image augmentation. The processing needs were lower because there were only a few feature extraction stages, but the performance fell short of expectations. The U-Net encoder is then replaced with ResNet and VGGNet, which are both pretrained with weights from ImageNet [50]. The dataset used to train the model was further expanded with image augmentation methods by Keras.  Table 1 and Table 2 summarise the performance of these models on the validation and test datasets. It is visible that the U-Net with VGG backbone and ImageNet pretrained weights achieved the highest performance.

Table 3 summarizes the performance of the U-Net model with VGG encoder on each of the 6 test images. The predicted segmentation on the test dataset is also visualized in Figure 4.

Many recent advances in the fields of machine learning and computer vision have been fueled by common benchmarks: models trained and tested on high-variance datasets that lend themselves well to powerful features [51]. Transfer learning allows you to take an existing model that has learnt very generalizable weights from a large dataset like ImageNet and fine-tune it to fit your specific use case. Convolutional networks are able to learn characteristics in a hierarchical order. As a result, the generic descriptors acquired from a ConvNet are a good place to start when fine-tuning existing models for a more specialized task.

The first experiment in our investigation was conducted on the U-Net, with weights starting at a random value. Nonetheless, the above results show that we achieve a little lower accuracy than the U-Net that uses ResNet and VGGNet to handle the encoder component, which is initialized with weights from the pretrained ImageNet. Despite a smaller training dataset, the absence of a random weight initialization bottleneck and an increase in the network's learning capacity could explain the improved performance. Compared to the ResNet backbone, we discovered that the U-Net model with VGGNet achieved the best results. VGG outperforms ResNet for image segmentation tasks, according to [52]. The VGG model was chosen as the fixed feature extractor baseline. The VGG has a simple architecture, with homogenous 3 × 3 convolution kernels and 2 × 2 maxpooling throughout the pipeline, which gives it an edge over other networks (which showed marginally superior results in some circumstances) [53]. With VGG as the backbone, the model's accuracy on test images ranged from 79.16% to 93.87%, with iOU ranging from 64.80% to 75.98%, F1 score ranging from 78.53% to 86.73%, Precision ranging from 81.20% to 92.15%, Recall rate ranging from 77.36% to 83.14%, and Dice coefficient ranging from 70.77% to 77.84%.

The article "Detecting Buildings and Nonbuildings from Satellite Images Using U-Net" was published in 2022. Journal: Comput Intell Neurosci.

A variety of augmentations, such as flipping, zoom in/zoom out, rotating, and shearing, can be used to improve the performance of the created model. The trained model's performance for building detection and segmentation can be improved by using these alternative augmentations during training. However, augmentation was done at random and only when the data batch was fed into the model to keep memory limitations to a minimum and to execute the existing and promising segmentation algorithm as efficiently as feasible. When photos with completely different features from those in the original training dataset appear in the real world, the diversified dataset will aid the model's generalization. When no development was noticed for more than 20 epochs, we deemed the training to be finished.  Figure 5 shows that training and validation were reduced with each epoch, showing that no overfitting occurred, owing in part to data augmentation. The Dice coefficient, the Accuracy of the training, and the validation datasets are likewise growing after each epoch and eventually stabilizing.

The training dataset is clearly unbalanced, as shown in Figure 6. It can be seen that pixels from the nonbuilding class dominate the dataset, accounting for 87.37% of the total, while pixels from the building class account for 12.62%.  Figure 7 shows the confusion matrix of image 2, where 32% of buildings are predicted as nonbuildings but only 1% of nonbuildings were predicted to be building classes. Despite the training dataset's imbalance, 68% of the pixels projected as buildings and 99% of the nonbuilding pixels overlap with the ground truth labels.

### 4.1. Comparative Analysis

Building recognition from satellite photos has been a significant, and difficult problem in recent decades as cities have developed significantly. Building extraction is computationally difficult due to its importance in many sectors. It is widely used in city planning and development, infrastructure development, urban mapping and management, marketing, and population estimation, among other things. It is critical to extract information from pictures in a consistent and reliable manner [54]. Detecting the building from satellite photographs with simply human effort, on the other hand, is time-consuming and inefficient [8, 54, 55]. As a result, using an automatic building detection method is required to resolve these challenges [8].

The article "Detecting Buildings and Nonbuildings from Satellite Images Using U-Net" was published in 2022. Journal: Comput Intell Neurosci.

Reference [43] used high-resolution satellite pictures from rural China to create the dataset for this investigation. The photos had a 0.26 m resolution. The images range in size from 900 × 900 to 1024 × 1024 pixels. The authors of this study attempted to develop the Mask R-CNN model, for developing instance segmentation. However, as part of our research, we created a semantic segmentation model that aids in the classification and segmentation of buildings in images, which also helps in various other tasks such as coverage estimation of the area's buildings and change detection.

We used a smaller number of training photos in our research. Other large datasets, such as Inria [56], contain data that are mislabeled or fuzzy. Furthermore, OSM users incorrectly defined the masks [56], which has a substantial impact on the model's performance.  Table 4 shows a few results from the literature that can be used to compare our findings. Reference [57] used the standard U-Net architecture, and the dataset was augmented. The dataset used was the SpaceNet building dataset provided in the CVPR 2018 DeepGlobe Satellite Challenge. However, the resolution is higher; as a result, there is a slight level of detail in the features of the classes that must be classified. The same dataset was utilized by [36]. Despite developing a novel model to handle the resolution of feature maps for small objects [36], they had trouble segmenting the small size buildings in the image.

Our model, which is based on a U-Net architecture with a VGG16 backbone that has been pretrained with ImageNet weights outperforms the other two. Model development was a faster and more efficient computing procedure with a smaller training dataset. It also demonstrates that our model can perform effectively on a limited number of examples, decreasing annotation time while maintaining segmentation capability.

## 5. Conclusions

The study attempted to segment all buildings in high-resolution satellite images automatically. The U-Net semantic segmentation model was proposed for this challenge since it provided the highest accuracy with the least amount of training data and processing power. We investigated the performance of the customized end-to-end U-Net model and the pretrained models in place of the encoder. According to the research, the pretrained models outperformed the state-of-the-art U-Net model because they were more robust in feature representation. The pretrained VGGNet encoder in the U-Net worked well in creating segmentation, attaining an Accuracy of 89.28%, iOU of 74.70%, F1 score 84.90%, Precision of 88.99%, Recall of 82.61%, and Dice score of 77.47% in an experiment on a tiny image dataset. According to the findings, the suggested U-Net considerably outperforms preceding models such as Mask R-CNN in terms of accuracy with limited training data. Future research aims to enlarge the training dataset and improve the network design to improve the suggested model's generalization capacity with a more extensive network and more processing power.

The article "Detecting Buildings and Nonbuildings from Satellite Images Using U-Net" was published in 2022. Journal: Comput Intell Neurosci.

## Figures and Tables

**Figure 1:** Sample images and corresponding ground truth masks (annotations) from the (a) training, (b) validation, and (c) test dataset.

**Figure 2:** U-Net architecture [21].

**Figure 3:** U-Net training and validation procedure.

**Figure 4:** Qualitative results on the test set.

**Figure 5:** Plots for Accuracy, Dice, loss, iOU segmentation loss, and MAE while training.

**Figure 6:** No. of pixels vs. classes in training, validation, and test datasets and predicted test set.

**Figure 7:** Confusion matrix of images from the test dataset.

**Table 1:** Performance of the various models on validation dataset.

Validation dataset	Trained models	Accuracy (%)	iOU (%)	F1 score (%)	Precision (%)	Recall (%)	Dice (%)
	U-Net with no augmentation	90.36	71.49	82.12	86.55	79.17	70.10
	U-Net with ResNet as backbone	90.88	72.37	82.77	88.44	79.34	71.15
	U-Net with VGG as backbone	92.58	77.44	86.57	89.85	84.09	77.79

**Table 2:** Performance of various models on test dataset.

Test dataset	Trained models	Accuracy (%)	iOU (%)	F1 score (%)	Precision (%)	Recall (%)	Dice (%)
	U-Net with no augmentation	87.78	70.91	82.08	88.98	78.99	72.64
	U-Net with ResNet as backbone	88.48	72.85	83.60	88.32	80.95	74.91
	U-Net with VGG as backbone	89.28	74.70	84.90	88.99	82.61	77.47

**Table 3:** Quantitative results on test images.

Images	Accuracy (%)	iOU (%)	F1 score (%)	Precision (%)	Recall (%)	Dice (%)
Image 1	90.40	74.03	84.24	91.49	80.30	74.38
Image 2	92.68	77.66	86.73	92.15	83.14	77.84
Image 3	93.87	75.07	84.50	91.85	79.91	72.46
Image 4	83.24	66.87	79.51	87.68	77.36	70.77
Image 5	79.16	64.80	78.53	81.20	78.53	74.86
Image 6	90.79	75.98	85.72	90.32	82.73	77.20

**Table 4:** Comparison with the previous works.

Ref	F1 score
[57]	**70.4**
[36]	**73.91**
**Ours**	**84.90**

## Data Availability

The dataset used in the study is extracted from the study by Li, Y.; Xu, W.; Chen, H.; Jiang, J.; Li, X; A Novel Framework Based on Mask R-CNN and Histogram Thresholding for Scalable Segmentation of New and Old Rural Buildings; *Remote Sens*. 2021, 13, 1070.
